The article "Dosimetric Comparison between Volumetric Modulated Arc Therapy (VMAT) and Intensity-Modulated Radiotherapy (IMRT) for Dental Structures of Head and Neck Cancer Patients" was retracted in 2022. Reason: concerns about the peer review.

# Dosimetric Comparison between Volumetric Modulated Arc Therapy (VMAT) and Intensity-Modulated Radiotherapy (IMRT) for Dental Structures of Head and Neck Cancer Patients

**DOI:** 10.1155/2022/4998997

**Published:** 2022-04-05

**Authors:** Yan Ma, Jianfeng Zhou, Hongyong Wang

**Affiliations:** ^1^Department of Radiation Oncology, The Second Hospital of Jilin University, Changchun 130041, Jilin, China; ^2^Department of Radiation Oncology, Shenzhen Hospital of Southern Medical University, Shenzhen, China

## Abstract

**Background:**

This retrospective study aimed to evaluate the radiation dose delivered to dental structures in intensity-modulated radiotherapy (IMRT) and volumetric modulated arc therapy (VMAT) without dental dose constraints, compare the dosimetry differences of dental structures between the two radiation techniques, and determine whether dental structures should be one of the organs at risk for IMRT and VMAT plans according to the dosimetric analysis.

**Materials and Methods:**

A total of 138 head and neck cancer patients (nasopharyngeal, oral cavity, pharyngeal, hypopharynx, and larynx), who underwent IMRT (69 patients) or VMAT (69 patients) from March 2016 to March 2021 in our hospital, were included to assess the dosimetry difference between two radiotherapy techniques for dental structures.

**Results:**

The radiation dose delivered by IMRT and the mean maximum doses delivered by VMAT to the maxillary teeth of nasopharyngeal cancer patients were significantly higher than the dose received by the mandibular teeth. In contrast, the mandibular teeth of oral cavity cancer, oropharynx cancer, and laryngeal cancer received higher radiation doses than maxillary teeth. Except for mandibular teeth of oral cancer patients, the molars received significantly high-dose radiation than premolars and/or incisors in both radiotherapy techniques. No significant difference was observed between IMRT and VMAT in the dosimetric comparison of dental structures, except that oral cavity cancer patients treated with VMAT received a significantly higher mean average dose than those treated with IMRT. When PTV included level Ib, the radiation doses of the mandibular teeth delivered by both radiotherapy techniques were significantly higher than that in PTV when level Ib was excluded.

**Conclusion:**

Without dental dose constraints, no major difference was observed between IMRT and VMAT plans in tooth dose distribution. We suggest that dental structures should be delineated as part of the organ at risk (OAR) when IMRT and VMAT are planned. Meanwhile, attention should be paid to dental structures that might have a high-dose area according to the specific tumor location.

The article "Dosimetric Comparison between Volumetric Modulated Arc Therapy (VMAT) and Intensity-Modulated Radiotherapy (IMRT) for Dental Structures of Head and Neck Cancer Patients" was retracted in 2022. Reason: concerns about the peer review.

## 1. Introduction

There were an estimated 931931 newly diagnosed head and neck cancers and 467125 relevant deaths worldwide in 2020, according to the GLOBOCAN estimates of cancer incidence and mortality produced by the International Agency for Research on Cancer [1]. Radiotherapy is one of the main treatment options for head and neck cancers. With the development of radiotherapy technology, the five-year survival rate of head and neck cancer (HNC) patients has improved [2–4]. However, radiation therapy is a double-edged sword, damaging normal tissues while killing tumors. Therefore, in the process of tumor treatment, how to better protect normal tissues has always been a problem that needs to be solved in radiotherapy. Most HNC patients have different symptoms and signs of periodontal diseases, such as gingival bleeding, periodontal pocket formation, gingival atrophy, loss of periodontal attachments, and tooth mobility during and after radiotherapy, significantly decreasing patients' quality of life [5–7]. High-dose radiation can directly damage dental structures and then develop into radiation-related caries (RRC) [8, 9]. Furthermore, RRC will increase the risk of tooth loss, seriously influencing the patient's quality of life [10, 11]. Therefore, dose constraints for dental structures during radiotherapy in HNC patients should become the focus of the whole treatment course. However, Radiation Therapy Oncology Group (RTOG) consensus contouring guidelines for head and neck OAR did not include dental structures. This might result in some radiation centers' decision not to use the dental structures as an OAR to limit radiation doses when formulating radiotherapy plans, and the dental structures might receive high radiation doses. In the present study, we evaluated radiation doses delivered to dental structures of IMRT and VMAT techniques without dental dose constraints of different HNC patients. We observed whether the radiotherapy dose is too high for the dental structures without dose constraints. And based on previous studies on the relationship between dental radiation dose and dental side effects of radiotherapy, we determined whether to use dental structures as part of the OAR of the IMRT and VMAT plan.

The quality of radiotherapy techniques is directly related to the efficacy of treatment and the quality of life because better radiotherapy technology can reduce the radiation dose of normal tissues as much as possible and at the same time can provide a higher radiation dose for the target area. Compared with 3D-conformal radiotherapy (3D-CRT), IMRT and VMAT can provide more conformal dose coverage for the treatment area, reduce the dose to the OAR, improve treatment efficacy, and reduce side effects [12–15]. IMRT was proposed by Kijewski et al. in the 1970s [16]. The 3D-CRT requirements specify that the shape of the radiation field in the radiation field direction must be consistent with the shape of the target volume. In addition, the output dose rate in each radiation field must be adjusted as required so that the dose on the surface of the target volume can be equal everywhere to achieve the 3D-conformal appropriate effect of the dose distribution. VMAT technique is a superposition of Arc therapy and IMRT technologies. VMAT technology refers to an intensity-modulated radiotherapy technology where the speed of the gantry, the angle of the collimator, the position of the multileaf collimator (MLC) leaf, and the dose rate can be continuously changed during the rotation of the accelerator frame to realize the modulation of the beam intensity at each position. The number of radiation arcs of VMAT can be single or more, and the quality of the VMAT plan is related to the complexity of the target volume and the number of arcs. Current research agrees that compared with IMRT, VMAT can reduce the treatment time and monitor units (MU) [17–20]. To the best of our knowledge, this is the first comprehensive study to evaluate the dosimetric distribution of dental structures delivered by VMAT and compare the exposure doses of dental structures without dose constraints of IMRT and VMAT.

The article "Dosimetric Comparison between Volumetric Modulated Arc Therapy (VMAT) and Intensity-Modulated Radiotherapy (IMRT) for Dental Structures of Head and Neck Cancer Patients" was retracted in 2022. Reason: concerns about the peer review.

This retrospective study aimed to (a) evaluate radiation doses received by dental structures in IMRT and VMAT techniques; (b) compare the dosimetry difference of dental structures between two radiation techniques without dental structure constraints; (c) determine whether dental structures should be one of the organs at risk for IMRT and VMAT plans according to the dosimetry analysis.

## 2. Material and Methods

### 2.1. Patients

First, we counted all HNC patients who received radiotherapy in our hospital from March 2016 to March 2021 and then adopted a stratified proportional sampling method to identify 138 HNC patients treated with IMRT or VMAT included in the present study. All the patients underwent pathological biopsies and enhanced MRI as the basis for staging, and cases with braces, metallic teeth, and other items affecting CT imaging or dose calculations were excluded. The tumor's stage was based on the American Joint Committee on *Cancer* (AJCC) staging system. The patients were divided into four groups of nasopharyngeal, oral cavity, pharyngeal, hypopharyngeal, and laryngeal cancers, according to tumor location. Informed consent was obtained from all patients and informed consent was signed during the experiment.

The article "Dosimetric Comparison between Volumetric Modulated Arc Therapy (VMAT) and Intensity-Modulated Radiotherapy (IMRT) for Dental Structures of Head and Neck Cancer Patients" was retracted in 2022. Reason: concerns about the peer review.

### 2.2. Treatment Planning

All the patients were fixed with a thermoplastic head–neck and shoulder mask in the supine position. The coverage of contrast-enhanced CT scan extended from the vertex to the clavicle using a 16-slice CT scanner (The Philips Brilliance CT Big Bore Oncology Configuration, Cleveland, OH) and reconstructed with a layer spacing of 3 mm. The gross tumor volume (GTV), clinical target volume (CTV), planning target volume (PTV), and OARs were delineated according to the guidelines of the International Commission on Radiation Units and Measurements (ICRU) 50/62 reports and the experience of our hospital. The target areas of radiotherapy for all the patients were completed by three experienced radiation oncologists of HNC in our hospital. Furthermore, due to personal habits, the naming of the target area is slightly different. Therefore, in the present research, to facilitate the statistics of the prescription dose, the treatment target area is named uniformly. Therefore, the GTV-T was uniformly defined as the primary tumor or tumor bed, and GTV-N was defined as imageological positive lymph nodes. Low-risk CTV and high-risk CTV were defined as CTV1 and CTV2, respectively. PGTVt and PGTVn were formed by expanding GTVt and GTVn 5 mm in various directions, respectively. PTV1 and PTV2 were defined as CTV1 and CTV2 plus a 5 mm margin.  Table 1 presents the mean prescription doses in the target area of different tumors. VMAT double-arc plan and 7–9 beam dynamic IMRT plan were achieved by radiotherapy physicists using the progressive resolution optimization in the Eclipse treatment planning system (version 10.0). All the patients were treated with 6-MV photon beams generated from Varian TrueBeam linear accelerator.

### 2.3. Delineation of Dental Structures

Two oral oncologists delineated the dental crowns of each patient with the assistance of two medical physicists. The dental crown was divided into maxillary and mandibular teeth during the delineating process, while the maxillary and mandibular teeth were further classified into three groups of incisors (anterior), premolars, and molars. After delineating, the cumulative dose of each group included the mean of maximum doses, and the mean of average doses was recorded. Also, the level I nodal region is the lymphatic drainage area closest to the dental crowns of mandibular teeth. The exposure dose of dental structures might be affected by whether PTV includes the area, especially in the molars group. We, therefore, identified patients in the PTV inclusion level I nodal region and compared them with patients in the PTV exclusion level I nodal region to investigate the difference in dose of the dental crowns between the two groups.

The article "Dosimetric Comparison between Volumetric Modulated Arc Therapy (VMAT) and Intensity-Modulated Radiotherapy (IMRT) for Dental Structures of Head and Neck Cancer Patients" was retracted in 2022. Reason: concerns about the peer review.

### 2.4. Statistical Analyses

Radiation doses received by dental structures were analyzed for normality (Shapiro-Wilk test) and homogeneity of variance (Levene's test). The data conforming to the normal distribution were represented as mean (± standard deviation [SD]), while shown as median (interquartile range [IQR]). The independent-samples *t*-test or one-way ANOVA with SNK-q test was used for the data meeting the normal distribution; otherwise, Mann-Whitney test or Kruskal-Wallis test was used. The difference was statistically significant with two-tail *p* < 0.05. Statistical analyses were performed on the data using SPSS (version 27.0; SPSS Inc., Chicago, IL).

## 3. Results

Table 2 presents the clinicopathological information, including age, gender, TNM (T, invasive depth; N, lymph node metastasis, and *M*, distant metastasis) stage of the patients and tumor locations. There were 69 patients in the IMRT group, with a mean age of 55 years. Meanwhile, the mean age of 69 patients in the VMAT group was 58 years. Eight patients in the IMRT group received radical radiotherapy, with five patients in the VMAT group. Sixty-one patients in the IMRT group underwent concurrent chemoradiotherapy, with 64 patients in the IMRT group.

### 3.1. Dosimetric Distribution to Dental Structures in IMRT

A comparison of the overall dental doses of different tumor locations treated with IMRT showed dental structures of patients with laryngeal cancer received lower radiation doses than other patients, and statistical significance was achieved with the mean of maximum doses (*p* < 0.001) (Figure 1(a)). Radiation doses delivered by IMRT to the maxillary and mandibular teeth were also compared. The maxillary teeth of nasopharyngeal cancer patients received significantly higher radiation doses than the mandibular teeth (average dose: *p* < 0.001; maximum doses: *p*=0.049). In contrast, mandibular teeth in the oral cavity, oropharyngeal, and laryngeal cancer patients received higher radiation doses than maxillary teeth; however, statistically significant differences were not found in the mean maximum doses in laryngeal cancers (*p*=0.20) (Table 3). Additionally, when assessing the maxillary or mandibular teeth of different tumor locations, we found that the maxillary teeth of patients with nasopharyngeal cancers received significantly higher radiation doses than the maxillary teeth of the other three groups (average and maximum doses: *p* < 0.001).

On the other hand, the mandibular teeth of oral cavity cancer patients received higher radiation doses than all the other patients, and statistical significance was achieved with the mean of average doses (*p* < 0.001). Meanwhile, the mean maximum dose of the mandibular teeth of patients with laryngeal cancer was significantly lower than that of other patients (*p* < 0.001) (Table 3). Thus, when it comes to evaluating the radiation dose received by patients in terms of tooth types at the same tumor location, we found that except for the mandibular molars of oral cavity cancer patients (average doses: *p*=0.616; maximum doses: *p*=0.164), the molars of other patients received significantly higher radiation doses than premolars and/or incisors (Table 4).

The article "Dosimetric Comparison between Volumetric Modulated Arc Therapy (VMAT) and Intensity-Modulated Radiotherapy (IMRT) for Dental Structures of Head and Neck Cancer Patients" was retracted in 2022. Reason: concerns about the peer review.

### 3.2. Dosimetric Distribution to Dental Structures in VMAT

The overall dental doses of different tumor locations treated with VMAT were also compared. The results showed that the mean of average radiation dose delivered by VMAT to patients with oral cavity cancers was significantly higher than other patients (*p* < 0.001). In addition, dental structures in patients with laryngeal cancer received significantly lower radiation doses than other patients (average and maximum doses: *p* < 0.001) (Figure 1(b)). By evaluating maxillary and mandibular tooth dosages according to primary tumor locations, we discovered that the mean maximum doses of maxillary teeth in nasopharyngeal cancer were significantly higher than mandibular teeth (*p*=0.04). In contrast, compared with the maxillary teeth, the mandibular teeth of patients with laryngeal, oral cavity, and oropharyngeal cancers received significantly higher radiation doses (Table 5). Similar to the results of the IMRT treatment group, in the maxillary or mandibular teeth of different tumor locations, VMAT delivered more radiation doses to the maxillary teeth of nasopharyngeal cancer patients than the upper teeth of other patients (average and maximum doses: *p* < 0.001). At the same time, the mandibular teeth of oral cavity cancer patients received higher doses than those affected by other cancers (average and maximum doses: *p* < 0.001) (Table 5). The same result was also found in the VMAT treatment group; that is, molars received significantly higher doses than premolars and/or incisors except for the mandibular molars of oral cavity cancer patients (average doses: *p*=0.77; maximum doses: *p*=0.386) (Table 4).

### 3.3. Comparison of Dosimetric Distribution between IMRT and VMAT

Radiation doses produced by IMRT and VMAT to the overall dental structures were also evaluated in the present study. We found that the radiation doses delivered by VMAT to overall dental structures were slightly higher than that of IMRT. However, there was no significant difference in the overall dental doses between IMRT and VMAT (average doses: *p*=0.33; maximum doses: *p*=0.947) (Figure 1(c)). When it referred to different tumor locations, we discovered that oral cavity cancer patients undergoing VMAT withstood significantly higher mean of average doses than those undergoing IMRT (*p*=0.04) (Figure 1(d)). However, no significant difference was found in the radiation doses delivered to maxillary teeth between IMRT and VMAT (average doses: *p*=0.772; maximum doses: *p*=0.843) (Figure 2(a)) and mandibular teeth (average doses: *p*=0.198; maximum doses: *p*=0.425) (Figure 2(b)).

The article "Dosimetric Comparison between Volumetric Modulated Arc Therapy (VMAT) and Intensity-Modulated Radiotherapy (IMRT) for Dental Structures of Head and Neck Cancer Patients" was retracted in 2022. Reason: concerns about the peer review.

### 3.4. Dosimetric Distribution to Dental Structures Related to Ib Level

The influence of delineation of level Ib on the dose distribution of tooth structures was also investigated in the present study. We found that when level Ib was delineated in the PTV, the radiation doses delivered to the mandibular teeth by IMRT and VMAT were significantly higher than that the PTV, excluding level Ib (IMRT: *p*=0.013 for average doses and *p*=0.003 for maximum doses; VMAT: *p*=0.023 for average doses and *p*=0.006 for maximum doses) (Figures 2(c) and 2(d)). In addition, when tooth types were considered, significant differences were also observed in the doses delivered by the two techniques to incisors, premolars, and molars of the lower teeth between PTV including the level Ib and PTV excluding the level Ib (Table 6).

## 4. Discussion

There are many oral sequelae caused by radiotherapy for patients with HNC. Radiation-related caries, rampant caries appearing 6 to 12 months after radiotherapy in patients with HNC, is one of the severe complications of head and neck radiotherapy. The clinical manifestation of radiation-related caries is the simultaneous occurrence of caries on multiple teeth in a short time, mainly in the cervical and incisal areas of teeth. The irradiated teeth initially start as enamel cracks, and at the same time, a large area of enamel demineralization appears on the tooth smooth surfaces. If the demineralized area is not treated in time, brownish cavities will appear, and finally, extensive dental destruction will occur, affecting the patient's masticatory function [21–24]. The mechanism of RRC includes two aspects: direct factors and indirect factors [25]. Concerning direct factors, radiation can lead to changes in the mechanical properties and chemical composition of teeth, directly destroying the enamel, dentin, and the dentinoenamel junction [8, 26, 27]. Although most people believe that direct factors play a significant role in forming radiation-related caries, direct damage to the teeth by radiation is still not negligible. Therefore, when preparing a radiotherapy plan for patients with head and neck tumors, in addition to protecting the normal tissues, such as the parotid gland, dental structures should also be considered part of the OAR to ensure that the radiation dose of tooth structures is not too high.

The article "Dosimetric Comparison between Volumetric Modulated Arc Therapy (VMAT) and Intensity-Modulated Radiotherapy (IMRT) for Dental Structures of Head and Neck Cancer Patients" was retracted in 2022. Reason: concerns about the peer review.

Previous studies have evaluated radiation doses of dental structures produced by 3D-CRT and IMRT but have not evaluate the radiation dose delivered to dental structures in VMAT without dental dose constraints comprehensively [28–32]. Our research addressed the limitations of previous studies. Walker et al. analyzed the relationship between the severity of dental lesions in 93 patients with HNC and the radiation doses received by the teeth. The results showed that when the radiation dose was <30 Gy, there was minimal tooth damage. When the radiation dose reached 30 to 60 Gy, the risk of tooth damage was 2–3 times higher than that of the nonirradiated teeth. In addition, compared with teeth not exposed to radiation, teeth with a dose >60 Gy were 10 times more likely to sustain tooth damage [33]. According to this study, when radiotherapy is performed on patients with head and neck tumors, it is necessary to ensure that the radiation dose to the teeth should be <60 Gy, preferably <30 Gy, to significantly reduce the risk of dental incidents. Therefore, we focused on areas where the dental structure was exposed to a dose of >30 Gy in the present study. We found that in two different radiotherapy techniques, the maxillary teeth of nasopharyngeal cancer patients received higher radiation doses than both the mandibular teeth of patients with nasopharyngeal cancer and the maxillary teeth of patients with other tumor locations. Meanwhile, the mean of maximum doses exceeded 60 Gy. By observing the dose data of different tooth types, we found that the high-dose area was located in the molars, consistent with a study by Parahyba et al. [28]. We also found that except for the mean of maximum doses of the mandibular anterior teeth with IMRT technology that was slightly <60 Gy, the radiation doses received by the other mandibular tooth types in oral cavity cancer patients in IMRT and VMAT exceeded 60 Gy. In addition, the mandibular molars of patients with oropharyngeal cancer are adjacent to the oropharyngeal and lymph node areas and are often included in the radiation field; the radiation dose in this area was >60 Gy in the present research. Therefore, when formulating the IMRT and VMAT plans, the dose constraints in this area should be considered. Furthermore, the radiation dose delivered by the two radiation techniques to the maxillary and mandibular teeth of patients with laryngeal cancer did not exceed 60 Gy, but it still exceeded 30 Gy because the PTV of patients with laryngeal cancer is relatively far from teeth compared with the other three types of HNC patients. In addition, compared with other tumor locations, more energy can be devoted to protecting other OAR, such as the parotid glands, which can help reduce the incidence of radiation-related caries. Finally, when level Ib was included in the PTV, the radiation dose delivered to mandibular teeth, especially the mandibular molars, was significantly higher than PTV excluding level Ib, consistent with a study by Polce et al. [31]. Furthermore, the radiation dose delivered to mandibular molars reaches or approaches 60 Gy using these two radiotherapy techniques. Therefore, it is necessary to focus on limiting the dose in the mandibular molar area when PTV includes level Ib. In summary, we hold that dental structures should also be limited as part of OAR when developing the IMRT and VMAT plan. Furthermore, for a specific patient with HNC undergoing radiotherapy, personalized dental dose limitation measures should be formulated.

The article "Dosimetric Comparison between Volumetric Modulated Arc Therapy (VMAT) and Intensity-Modulated Radiotherapy (IMRT) for Dental Structures of Head and Neck Cancer Patients" was retracted in 2022. Reason: concerns about the peer review.

Some studies have evaluated the VMAT and IMRT plans for patients with head and neck cancers [17, 34–36]. These studies have compared the dosimetric difference of VMAT plans with different numbers of arcs and IMRT plans with different beam numbers and beam angles. In terms of the ability to spare OAR, the consensus view of these studies is that VMAT is equal to or slightly superior to IMRT. The present research compared the dose distribution of dental structures of IMRT and VMAT with no dental constraints. The results showed no apparent differences in dental structure dose distribution between the IMRT and VMAT plans in the four common head and neck tumors. However, to the best of our knowledge, no research is available on comparing the difference in dental structure dose distribution between these two radiotherapy techniques under the condition of limited tooth dose. Therefore, future research can be devoted to this aspect to better protect tooth structures during radiotherapy and reduce the risk of adverse dental events. Concerning limited tooth dose, the pros and cons of the two radiotherapy techniques for tooth protection should be evaluated in future studies.

## 5. Conclusion

In our opinion, regardless of the IMRT plan or the VMAT plan, dental structures should be delineated as part of the OAR. At the same time, attention should be paid to dental structures that might have a high-dose area according to the specific tumor location to limit the radiation dose to dental structures within an acceptable range. By referring to the studies of other scholars, the radiation dose used in this study was controlled between 30 and 60 Gy, and the research effect was good. The radiation dose used in this study can provide dose reference for oral cancer patients in clinical radiotherapy. In the present study, no significant difference was observed between IMRT and VMAT plans in tooth dose distribution without limiting the dose of dental structures.

The article "Dosimetric Comparison between Volumetric Modulated Arc Therapy (VMAT) and Intensity-Modulated Radiotherapy (IMRT) for Dental Structures of Head and Neck Cancer Patients" was retracted in 2022. Reason: concerns about the peer review.

## Figures and Tables

**Figure 1:** Radiation doses delivered by IMRT and VMAT to the overall dental structures. N independent-samples *t*-test or one-way ANOVA was used to compare radiation doses (*p* < 0.05). (a) The dental structure of patients with laryngeal cancer undergoing IMRT received lower radiation doses than other patients, and statistical significance was achieved with the mean of maximum doses. Mean of average doses: nasopharynx: 34.53 ± 3.01 Gy, oral cavity: 35.79 ± 11.39 Gy, oropharynx: 29.27 ± 10.88 Gy, and larynx: 25.08 ± 6.86 Gy. Mean of maximum doses: nasopharynx: 66.99 ± 6.72 Gy, oral cavity: 63.87 ± 9.17 Gy, oropharynx: 61.72 ± 9.27 Gy, and larynx: 45.77 ± 11.41 Gy. (b) The mean of average radiation doses delivered by VMAT to patients with oral cavity cancers was significantly higher than other patients. In addition, the dental structures of patients with laryngeal cancers received significantly lower radiation doses than other patients. Mean of average doses: nasopharynx: 34.25 ± 5.24 Gy, oral cavity: 43.02 ± 10.79 Gy, oropharynx: 30.20 ± 11.78 Gy, and larynx: 23.57 ± 6.30 Gy. Mean of maximum doses: nasopharynx: 63.62 ± 7.82 Gy, oral cavity: 65.47 ± 10.72 Gy, oropharynx: 61.72 ± 9.27 Gy, and larynx: 46.69 ± 10.76 Gy. (c) There were no significant differences in the overall dental doses between IMRT and VMAT. Mean of average doses: IMRT: 30.93 ± 9.49 Gy; VMAT: 32.84 ± 11.14 Gy. Mean of maximum doses: IMRT: 59.47 ± 12.32 Gy; VMAT: 59.61 ± 12.31 Gy. (d) Patients affected by oral cavity cancers treated with VMAT received significantly higher means of average doses than those treated with IMRT. Mean of average doses: IMRT: 35.79 ± 11.39 Gy; VMAT: 43.68 ± 10.79 Gy. Mean of maximum doses: IMRT: 63.87 ± 9.17 Gy; VMAT: 64.84 ± 10.13 Gy.

**Figure 2:** The radiation doses of maxillary and/or mandibular teeth delivered by IMRT and VMAT. Independent-samples *t*-test was used to compare radiation doses (*p* < 0.05). (a) No significant differences were found in the radiation doses between IMRT and VMAT to the maxillary teeth. Mean of average doses: IMRT: 26.98 ± 11.22 Gy; VMAT: 30.11 ± 8.53 Gy. Mean of maximum doses: IMRT: 49.48 ± 16.97 Gy; VMAT: 50.08 ± 18.98 Gy. (b) No significant differences were found in the radiation doses between IMRT and VMAT to the mandibular teeth. Mean of average doses: IMRT: 35.27 ± 11.90 Gy; VMAT: 38.11 ± 13.97 Gy. Mean of maximum doses: IMRT: 56.01 ± 11.80 Gy; VMAT: 57.64 ± 12.25 Gy. (c) The means of average and maximum doses of the mandibular teeth delivered by IMRT were significantly higher than when PTV excluded level Ib. Mean of average doses: PTV included level Ib: 37.63 ± 12.54 Gy; PTV excluded level Ib: 30.11 ± 8.53 Gy. Mean of maximum doses: PTV included level Ib: 58.77 ± 11.03 Gy; PTV excluded level Ib: 49.98 ± 11.39 Gy. (d) The means of average and maximum doses of the lower teeth delivered by VMAT were significantly higher than the PTV excluding level Ib. Mean of average doses: PTV included level Ib: 40.62 ± 15.01 Gy; PTV excluded level Ib: 32.38 ± 9.18 Gy. Mean of maximum doses: PTV included level Ib: 60.30 ± 11.66 Gy; PTV excluded level Ib: 51.57 ± 11.63 Gy.

The article "Dosimetric Comparison between Volumetric Modulated Arc Therapy (VMAT) and Intensity-Modulated Radiotherapy (IMRT) for Dental Structures of Head and Neck Cancer Patients" was retracted in 2022. Reason: concerns about the peer review.

**Table 1:** The prescribed doses to the target area of different tumor locations delivered by IMRT and VMAT.

		Nasopharynx	Oral cavity	Oropharynx	Larynx
IMRT	PGTV	73.02 ± 0.98	65.86 ± 5.49	65.11 ± 9.97	67.31 ± 10.60
	PGTVn	67.97 ± 2.28	66.17 ± 2.56	63.04 ± 8.31	69.03 ± 7.17
	PTV	65.8 ± 1.82	60.65 ± 5.0	57.07 ± 5.87	63.11 ± 6.71

VMAT	PGTV	75.46 ± 1.13	68.87 ± 6.53	70.42 ± 5.34	72.25 ± 5.26
	PGTVn	72.53 ± 2.02	66.23 ± 4.9	68.82 ± 4.11	66.93 ± 4.11
	PTV	66.0 ± 1.97	62.91 ± 5.45	63.15 ± 5.28	62.85 ± 4.38

**Table 2:** The clinicopathological data of HNC patients.

Characteristics	No. of patients (%)	
	IMRT (*n* = 69)	VMAT (*n* = 69)
Tumor location		
Nasopharynx	18 (26.1%)	18 (26.1%)
Oral cavity	17 (24.6%)	17 (24.6%)
Oropharynx	16 (23.2%)	16 (23.2%)
Larynx	18 (26.1%)	18 (26.1%)

T classification		
T1	12 (17.4%)	8 (11.6%)
T2	33 (47.8%)	25 (36.2%)
T3	11 (15.9%)	23 (33.3%)
T4	13 (18.9%)	13 (18.9%)

N classification		
N0	30 (43.5%)	20 (29.0%)
N1	13 (18.8%)	13 (18.8%)
N2	25 (36.2%)	32 (46.4%)
N3	1 (1.5%)	4 (5.8%)

M classification		
M0	69 (100%)	69 (100%)
M1	0 (0.0%)	0 (0.0%)

Age		
Mean	55	58
Range	16–70	16–87

Sex		
Male	50 (72.5%)	62 (89.9%)
Female	19 (27.5%)	7 (10.1%)

**Table 3:** Radiation doses received by maxillary and mandibular teeth using IMRT.

		Nasopharynx	Oral cavity	Oropharynx	Larynx
Maxillary teeth	Mean of average	37.56 ± 3.46 ^aA^	24.60 ± 11.41 ^bA^	23.22 ± 12.3 ^bA^	22.21 ± 8.46 ^bA^
	Mean of maximum	67.00 ± 6.72 ^aA^	45.66 ± 3.48 ^bA^	46.29 ± 16.8 ^bA^	38.57 ± 14.50 ^bA^

Mandibular teeth	Mean of average	31.49 ± 3.93 ^aB^	49.76(7.34)^bB^	35.31 ± 11.45 ^aB^	27.95 ± 6.05 ^aB^
	Mean of maximum	54.77 ± 6.65 ^aB^	63.87 ± 9.17 ^bB^	61.53 ± 9.28 ^bB^	42.34(10.70)^cA^

Different lowercase letters in the rows represent significant differences (*p* < 0.05) (one-way ANOVA or the Kruskal-Wallis test). In each row, we compared the radiation doses of maxillary and mandibular at different tumor locations. Different capital letters in the columns represent significant differences (*p* < 0.05) (independent-samples *t*-test or Mann-Whitney test). In each column, we compared the average doses (maximum dose) of the upper and lower teeth of the same tumor locations.

The article "Dosimetric Comparison between Volumetric Modulated Arc Therapy (VMAT) and Intensity-Modulated Radiotherapy (IMRT) for Dental Structures of Head and Neck Cancer Patients" was retracted in 2022. Reason: concerns about the peer review.

**Table 4:** Mean of the average and the maximum dosages received by tooth types of HNC patients.

		IMRT		VMAT	
		Mean (median) average	Mean (median) maximum	Mean (median) average	Mean (median) maximum
Nasopharynx	Mandibular teeth				
	Anterior teeth	22.09 ± 3.38^a^	31.26 ± 5.63^a^	26.60 ± 6.87^a^	31.65 ± 7.19^a^
	Premolars	29.12 ± 4.86^b^	36.27 ± 4.59^b^	31.31(6.06)^a^	38.23 ± 7.56^b^
	Molars	38.22 ± 5.33c	54.29 ± 6.76c	40.10 ± 6.52^b^	56.65 ± 8.68c
	Maxillary teeth				
	Anterior teeth	27.73 ± 4.61^a^	38.05 ± 5.89^a^	25.88 ± 7.19^a^	34.44 ± 8.16^a^
	Premolars	35.86 ± 4.12^b^	43.11 ± 5.13^b^	31.88 ± 7.06^b^	40.32 ± 7.35^b^
	Molars	45.20 ± 4.82^c^	66.23 ± 8.11^c^	43.51 ± 5.51^c^	63.84 ± 6.55^c^

Oral cavity	Mandibular teeth				
	Anterior teeth	48.87(15.00)^a^	59.60(15.82)^a^	52.04 ± 13.57^a^	61.39 ± 12.76^a^
	Premolars	51.04(8.64)^a^	61.83(12.19)^a^	54.03 ± 12.62^a^	63.72 ± 11.72^a^
	Molars	52.83(16.53)^a^	63.44 ± 8.92^a^	55.01 ± 11.39^a^	63.25(15.25)^a^
	Maxillary teeth				
	Anterior teeth	18.91 ± 8.67^a^	30.06 ± 10.21^a^	25.88 ± 12.85^a^	34.77 ± 13.94^a^
	Premolars	23.89 ± 11.54^a^b	34.04 ± 11.35^a^	29.54 ± 12.70^a^	41.35 ± 15.28^a^
	Molars	29.16 ± 13.97^b^	45.47 ± 13.37^b^	35.88 ± 14.01^b^	53.13 ± 14.87^b^

Oropharynx	Mandibular teeth				
	Anterior teeth	26.21 ± 11.40^a^	37.16 ± 15.20^a^	27.93 ± 13.68^a^	35.61 ± 17.15^a^
	Premolars	34.44 ± 14.14^a^	44.99 ± 12.39^a^	30.35(20.50)^a^	44.60 ± 15.11^a^
	Molars	43.08 ± 11.64^b^	62.18 ± 9.47^b^	42.82 ± 11.17^b^	61.90 ± 10.66^b^
	Maxillary teeth				
	Anterior teeth	15.88 ± 8.42^a^	24.39 ± 13.92^a^	18.92 ± 12.59^a^	27.75 ± 19.60^a^
	Premolars	21.16 ± 12.97^ab^	29.16 ± 13.75^a^	22.51 ± 15.31^a^	31.17 ± 17.84^a^
	Molars	29.11 ± 15.06^b^	45.20 ± 16.92^b^	30.83 ± 19.36^b^	47.50 ± 22.89^b^

Larynx	Mandibular teeth				
	Anterior teeth	20.45 ± 5.22^a^	29.68 ± 6.46^a^	20.34(11.67)^a^	27.27(12.10)^a^
	Premolars	26.68 ± 6.71^b^	33.26 ± 5.96^a^	23.77(8.70)^a^	32.03 ± 9.99^a^
	Molars	32.34 ± 6.91^c^	44.32 ± 11.60^b^	32.00 ± 8.27^b^	46.00 ± 11.02^b^
	Maxillary teeth				
	Anterior teeth	17.49 ± 6.73^a^	24.44 ± 9.66^a^	15.31 ± 7.59^a^	19.71(13.20)^a^
	Premolars	20.21 ± 8.92^ab^	27.42 ± 10.44^a^	17.79 ± 8.35^ab^	22.37 ± 9.32^a^
	Molars	25.69 ± 9.46^b^	37.98 ± 14.59^b^	22.28 ± 9.61^b^	32.54 ± 13.50^b^

Different lowercase letters in the columns represent significant differences (*p* < 0.05) (one-way ANOVA or the Kruskal-Wallis test). In each column, we compared tooth types of mandibular teeth (maxillary teeth) themselves.

The article "Dosimetric Comparison between Volumetric Modulated Arc Therapy (VMAT) and Intensity-Modulated Radiotherapy (IMRT) for Dental Structures of Head and Neck Cancer Patients" was retracted in 2022. Reason: concerns about the peer review.

**Table 5:** Radiation doses received by maxillary and mandibular teeth using VMAT.

		Nasopharynx	Oral cavity	Oropharynx	Larynx
Maxillary teeth	Mean of average	35.30 ± 5.75 ^aA^	31.56 ± 12.78 ^abA^	19.45(22.44) ^bcA^	18.89 ± 8.30^cA^
	Mean of maximum	64.73 ± 6.31 ^aA^	54.57 ± 14.49 ^abA^	48.03 ± 22.81 ^bA^	33.80(15.82)^cA^

Mandibular teeth	Mean of average	35.84(7.55) ^aA^	54.49 ± 12.68 ^bB^	33.73(20.46) ^aB^	27.61(6.68)^aB^
	Mean of maximum	57.06 ± 8.76 ^aB^	65.46 ± 10.72^bB^	62.36 ± 10.53^bcB^	46.36 ± 10.36^bB^

Different lowercase letters in the rows represent significant differences (*p* < 0.05) (one-way ANOVA or the Kruskal-Wallis test). In each row, we compared the radiation doses of maxillary and mandibular teeth of different tumor locations. Different capital letters in the columns represent significant differences (*p* < 0.05) (independent-samples *t*-test or Mann-Whitney test). In each column, we compared the average doses (maximum dose) of the upper and lower teeth of the same tumor locations.

**Table 6:** Mean of the average and the maximum dosages delivered to dental structures by IMRT and VMAT according to whether PTV included level Ib or not.

		IMRT		VMAT	
		Mean (median) average	Mean (median) maximum	Mean (median) average	Mean (median) maximum
Anterior teeth	Include level Ib	30.50 ± 14.56^a^	41.22 ± 16.05^a^	34.87 ± 17.80^a^	42.04 ± 19.21^a^
	Exclude level Ib	21.45 ± 7.89^b^	30.48 ± 10.34^b^	26.13 ± 8.55^b^	31.85 ± 11.84^b^

Premolars	Include level Ib	36.93 ± 14.26^a^	46.20 ± 14.55^a^	38.33 ± 16.27^a^	47.90 ± 16.60^a^
	Exclude level Ib	28.02 ± 9.66^b^	35.50 ± 9.12^b^	29.42 ± 10.05^b^	36.30 ± 12.11^b^

Molars	Include level Ib	42.27 ± 12.18^a^	58.73 ± 11.14^a^	44.80 ± 12.71^a^	60.32 ± 11.29^a^
	Exclude level Ib	35.72 ± 9.09^b^	49.94 ± 11.36^b^	36.57 ± 9.99^b^	51.01 ± 12.28^b^

Different lowercase letters in the columns represent significant differences (*p* < 0.05) (independent-samples *t*-test). In each column, we compared the inclusion and exclusion of level Ib in the same tooth type.

## Data Availability

The datasets used and/or analyzed during the current study are available from the corresponding author on reasonable request.
